The article "Neuroprotective Effect of Moxibustion on Cerebral Ischemia/Reperfusion Injury in Rats by Downregulating NR2B Expression" was published in 2021. Journal: Evid Based Complement Alternat Med.

# Neuroprotective Effect of Moxibustion on Cerebral Ischemia/Reperfusion Injury in Rats by Downregulating NR2B Expression

**DOI:** 10.1155/2021/5370214

**Published:** 2021-10-25

**Authors:** Zhong Di, Qin Guo, Quanai Zhang

**Affiliations:** ^1^Department of Acupuncture and Moxibustion, The Third Affiliated Hospital of Zhejiang Chinese Medical University, Hangzhou, China; ^2^Department of Acupuncture and Moxibustion, The Third School of Clinical Medicine, Zhejiang Chinese Medical University, Hangzhou, China

## Abstract

**Objective:**

Stroke is a common and frequently occurring disease of the central nervous system, which is characterized by high mortality and a high disability rate. Moxibustion is a common method for treating stroke in traditional Chinese medicine, but its neuroprotective mechanism is unknown. N-Methyl-D-Aspartate Receptor Subunit 2B (NR2B) plays an important role in neuronal apoptosis. The objective of this study was to explore the mechanisms underlying the neuroprotective effect of moxibustion on cerebral ischemia/reperfusion (I/R) injury based on NR2B.

**Methods:**

Sprague–Dawley rats were randomly divided into 5 groups: the control group, I/R group, I/R + moxibustion group, I/R + Ro25-6981 (NR2B antagonist) group, and I/R + Ro25-6981 + moxibustion group. The cerebral ischemia/reperfusion model was induced by middle cerebral artery occlusion. Before the establishment of the model, the Ro25-6981 group received intraperitoneal injections of Ro25-6981, the moxibustion group received moxibustion, and the Ro25-6981 + moxibustion group received both interventions. The neurological dysfunction was evaluated by a neurological deficiency score (NDS). The infarct volume was examined by TTC (2,3,5-triphenyltetrazolium chloride) staining. The apoptosis rate of cerebral cells in the ischemic area was examined by TUNEL (terminal deoxynucleotidyl transferase-mediated dUTP nick end labeling) staining, and the expression of Bcl-2, Bax, and caspase-3 was observed by western blot. NR2B and JNK were also observed by western blot.

**Results:**

Compared with the I/R group, moxibustion significantly decreased the neurological deficiency score (*P* < 0.05) and the infarct rate (*P* < 0.01) in I/R rats which were similar to those in the Ro25-6981 group. After moxibustion treatment, there was a significant decrease in the apoptosis rate (*P* < 0.001) and the protein expression levels of Bax, caspase-3, and JNK (*P* < 0.001) and an increase in the expression of Bcl-2 (*P* < 0.01). Compared with the I/R group, moxibustion downregulated the expression of NR2B and decreased the activity of NR2B in the cerebral ischemia area (*P* < 0.001).

**Conclusions:**

Moxibustion can improve neurological dysfunction and decrease infarction area and neuronal apoptosis caused by cerebral ischemia/reperfusion in rats. Its neuroprotective mechanism may be related to downregulating the expression of NR2B.

## 1. Introduction

Stroke has a high mortality and disability rate [1, 2] and imposes huge economic burdens worldwide [3]. Among the types of stroke, ischemic stroke accounts for approximately 87% of cases [4]. Ischemia/reperfusion injury caused by cerebral ischemia or recanalization is an important cause of neurological deficits and neuronal apoptosis [5]. Cerebral ischemia/reperfusion injury involves a series of complex pathophysiological events, including inflammation, oxidative stress, abnormal energy metabolism, and synaptic and extrasynaptic glutamate accumulation, resulting in nerve cell death and neurological impairment. The important role of overactivated glutamate receptors, especially NMDA receptors, in cerebral ischemia/reperfusion injury has attracted wide attention [6, 7].

NMDA receptors are one of the three ionic receptors that mediate synaptic plasticity and contain multiple regulatory subunits [8]. Among these subunits, NR2A and NR2B are considered to be the most important components of functional NMDA receptor ion channels. Because of the widespread expression of NR2A and NR2B in the brain, these subunits have received the most extensive research. NR2A and NR2B play opposite roles in regulating synaptic plasticity or neuronal survival and apoptosis [9, 10] and have different relationships with neuronal death and ischemic tolerance in the ischemic area [11]. Previous studies have shown that NR2B is more likely to promote neuronal death [12], while NR2A is beneficial for neuroprotection [9]. Therefore, it is critical to intervene with the NR2B receptor to reduce apoptosis caused by cerebral ischemia/reperfusion.

Inhibiting the NR2B-related neuronal apoptosis pathway through NR2B antagonists is a good choice. In many animal models of cerebral ischemia, NR2B antagonists, including ifenprodil, eliprodil, CP-101606, and Ro25-6981 [13], showed good neuroprotective effects. Fischer et al. performed electrophysiological experiments, toxicity experiments, intracellular Na^+^, Ca^+^ determination, and other experiments and showed that compared with ifenprodil, Ro25-6981 exhibited a better inhibitory effect [14]. Ro25-6981 is an activity-dependent, voltage-dependent, and noncompetitive antagonist of NR2B [15]. Preconditioning or postprocessing of NR2B antagonists can induce a protective effect on cerebral inflammation [16]. Ro25-6981 preconditioning could significantly increase the number of Bcl-2 cells and decrease the number of Bax cells in the brains of ischemic-hypoxic rats, reduce the death of hypoxic-ischemic cells, and enhance neuroprotective effects [17, 18].

Modern studies have shown that moxibustion has good protective effects on the brain and can reduce the inflammatory reaction and neuronal apoptosis induced by ischemia and hypoxia by reducing the synthesis and release of CO [19], increasing the activity of endogenous antioxidant enzymes [20], and inhibiting the activity of nitric oxide synthase [21]. In a rat model of middle cerebral artery occlusion (MCAO) induced cerebral ischemia, moxibustion could reduce the expression of caspase-9, caspase-3, and Bax and increase the expression of Bcl-2 in ischemic brain tissue to reduce the inflammatory reaction and neuronal apoptosis induced by ischemia and hypoxia [22, 23]. Moxibustion, as a nondrug therapy, can be combined with Ro25-6981 to reduce brain injury caused by cerebral ischemia/reperfusion and enhance neuroprotective effects, which is the starting point of this study.

In this study, the improved thread occlusion method was used to establish a rat model of middle cerebral artery occlusion. By comparing the effects of moxibustion and Ro25-6981 plus moxibustion on NR2B, JNK, Bax, Bcl-2, and caspase-3 in the cerebral ischemic area, we explored the neuroprotective effect of moxibustion on cerebral ischemia/reperfusion (I/R) injury and its possible mechanism.

## 2. Methods

### 2.1. Experimental Animals

Adult male Sprague Dawley rats weighing 200–220 g were obtained from the Animal Research Center of Zhejiang University of Traditional Chinese Medicine. Before further experiments, the rats were adapted to the new environment (room temperature: 23 ± 2°C; relative humidity: 45 ± 15%; light condition: 8 : 00 in the morning, light-dark cycle for 12 hours) for one week. The animals were kept in sterile propylene cages with aseptic shells, the shells were changed every day, and the rats received free water and food. All procedures in this study followed the guidelines for laboratory care and the use of animals at the National Institutes of Health. All the experimental methods were approved by the Animal Use and Nursing Committee of the Animal Research Center of Zhejiang University of Traditional Chinese Medicine. The research program and animal care followed the committee's guidelines.

### 2.2. Groups and Interventions

Eighty male SD rats were randomly divided into five groups: control group (*n* = 16), I/R group (*n* = 16), I/R + moxibustion group (*n* = 16), I/R + Ro25-6981 group (*n* = 16), and I/R + Ro25-6981 + moxibustion group (*n* = 16). The hair of the acupoint area was removed before treatment. In the I/R + moxibustion group and the I/R + Ro25-6981 + moxibustion group, the rats were fixed and treated with moxibustion. Rats in the other groups only underwent grasping stimulation.

Point selection was as follows: Baihui (GV 20), located at the top of the head near the midpoint of the line between the apex of the two ears, and Dazhui (GV 14), the posterior center between the 7^th^ cervical vertebra and the first thoracic vertebra.

Moxibustion was performed on fixed rats. Vaseline was applied to the point at which the hair was removed. Moxa strips with diameters of 4 mm were prepared. Light one end of the moxa strips. The ignition end of moxibustion was suspended at approximately 2 cm above the selected acupoint [24]. GV 20 was treated first, followed by GV 14. Moxibustion at each acupoint was performed for 15 minutes. Moxibustion treatment began 3 days before model induction and was performed once a day for 3 consecutive days.

Animals in the I/R + Ro25-6981 + moxibustion group and the I/R + Ro25-6981 group were given Ro25-6981 (5.0 mg/kg) (Sigma, R7150) dissolved in saline through the abdominal cavity (I.P.) [17]. The drug was given three times at intervals of 24 hours. Rats in the control group, ischemic model group, and moxibustion group were given the same amount of normal saline (1.0 ml/kg). The time and frequency of administration were the same as those in the Ro25-6981 group.

### 2.3. Animal Models

The cerebral ischemia model was established by middle cerebral artery occlusion (MCAO) [25]. The rats were anesthetized by intraperitoneal injection with sodium pentobarbital (40 mg/kg), the depth of anesthesia was evaluated by severe pain, and the rats had a slight reaction. In brief, after cervical skin preparation, a surgical incision was performed on the right neck. The right common carotid artery (CCA), external carotid artery (ECA), and internal carotid artery (ICA) were separated. The proximal end of the ECA was cut and a nylon filament was inserted into the lumen of the ICA to block the origin of the middle cerebral artery (MCA). The average insertion depth of the thread occlusion was 18.5 ± 0.5 mm. After 2 hours, the thread was removed to establish reperfusion. In the control group, the operation procedure was the same as that in the I/R group, but no thread bolt was inserted, and the skin was sutured after disinfection.

Two hours after reperfusion, the neurological deficiency of rats was measured according to Zea Longa's scale [26]. Only animals with a score of 1 to 3 were considered successful.

### 2.4. Neurological Deficiency Score

The neurological deficiency score (NDS) was blindly evaluated at 6 h and 24 h after reperfusion. The NDS was based on a previously published scale [26] as follows: 0, no neurological deficit; 1, mild focal neurological deficit; 2, moderate focal neurological deficit; 3, severe focal deficit; and 4, lost consciousness or died. Only the animals with NDS of 1 to 3 at 2h after reperfusion were used in this study.

### 2.5. TTC Staining Measurement of the Infarct Region

Twenty-four hours after the operation, the animals were deeply anesthetized by an intraperitoneal injection of sodium pentobarbital (40 mg/kg). The rat brains were removed quickly and were sliced into 2.0 mm sections. TTC (1% w/V, Sigma, T8877) was prepared in PBS and water at 37°C until the TTC was dissolved. The slices were immersed in 10 ml of TTC solution and incubated at 37°C for 10 minutes. After TTC staining, normal tissue was red, and infarcted tissue was white. The infarct volume was measured by Image-Pro Plus 6.0. The infarct rate was calculated as follows: corrected infarct volume (%) = (contralateral hemispheric volume-ipsilateral noninfarct volume)/contralateral hemispheric volume × 100%.

### 2.6. TUNEL Staining to Detect Apoptosis in Rat Brains

The rat brain tissue was washed. Different concentrations of ethanol (50%, 70%, 85%, and 95% to anhydrous ethanol) were used to gradually dehydrate the tissue for 2 hours per stage. The tissue mass was made transparent, waxed, and embedded. Then, the tissue was sectioned to a thickness of 4–7 *μ*m. The slices were dewaxed with xylene I for 10 minutes and xylene II for 10 minutes. The dewaxed slices were treated with 100% ethanol, 95% ethanol, 85% ethanol, 75% ethanol, and double-distilled water for 3 minutes each. Prepare TUNEL reaction solution (Beyotime, c1088) and add it to the sample. The antiquenching seals and DAPI (1 : 500 diluted) seals were stored at −20°C and photographed by fluorescence microscopy. The relevant parts of the samples were collected and analyzed by microscopy, and the apoptosis rate was calculated.

### 2.7. Western Blot Analysis

Appropriate amounts of rat brain tissue were lysed and homogenized, and the supernatant was collected. After SDS-PAGE, the proteins were transferred to NC membranes. The NC membrane was sealed with 5% skimmed milk powder. The membrane was incubated with the following primary antibodies in Tris-buffered saline plus Tween (TBST) at pH 7.4 overnight at 4°C : GAPDH (D16H11) XP Rabbit mAb (1 : 1000, CST, 5174), cleaved caspase-3 (1 : 1000, Affinity, AF7022), Bax/Bcl-2 (1 : 1000, Affinity, AF0120), JNK (1 : 1000, Affinity, AF6319), and p-JNK (1 : 1000, Affinity, AF3320). Sheep anti-rabbit HRP-labeled secondary antibody (1 : 1000, Beyotime, A0208) was diluted with a blocking solution containing 5% skimmed milk. The reaction proceeded for 2 hours at room temperature. After the secondary antibody reaction, the secondary antibody was recovered. Then, the membrane was washed with TBST 5–10 min 3 times. After ECL chemiluminescence treatment, the images were scanned by a Tanon-5200 imaging system.

### 2.8. Statistical Analysis

IBM SPSS 20.0 was used for statistical analysis. The data used in the figures are presented as the means ± standard error of the mean (mean ± SEM). Differences between multiple groups were compared by one-way analysis of variance (ANOVA). A paired *t*-test was used to compare the differences between the two groups. A value of *P* < 0.05 indicated that there was a difference in the comparison.

## 3. Results

### 3.1. Moxibustion Alleviated Neurological Deficits

Cerebral I/R injury led to disorders of neurological function, such as sensory and motor dysfunction. The NDS was evaluated according to the scoring criteria of Zea Longa. The higher the score, the more severe the dysfunction. The control group had no neurological deficit. Compared with the control group, the I/R group had obvious neurological deficits (*P* < 0.05). At 6 h after reperfusion, the NDS was not significantly different between the groups except for the control group. At 24 h after reperfusion, the NDS of I/R + moxibustion group was significantly lower compared with the I/R group (*P* < 0.05), and the I/R + Ro25-6981 group and I/R + Ro25-6981 + moxibustion group had similar results (Figure 1).

Figure 1 shows the neurological deficit score in each group. The higher the score, the more severe the dysfunction. *∗∗∗P* < 0.001 compared to the control group; ^#^*P* < 0.05 versus the I/R group.

### 3.2. Moxibustion Reduced the Brain Infarction

Due to the loss of dehydrogenase activity in the ischemic area, the TTC staining was pale, while normal tissue was crimson. As shown in Figure 2, the brain tissue in the control group was normal, and all the sections of each layer of brain tissue were dark red and infarcted; after ischemia/reperfusion in the I/R group, the color of the brain tissue on the nonischemic side was dark red, and the sections of each layer of brain tissue on the ischemic side showed pale areas of different sizes.

Compared with those in the I/R group, after I/R + moxibustion treatment, the pale area, total volume, and infarction rates of ischemic lateral brain tissue were decreased (*P* < 0.01). Compared with I/R + Ro25-6981, after treatment with Ro25-6981 plus moxibustion, the pale area in each layer of ischemic brain tissue was significantly reduced, and the infarction rate was significantly decreased (*P* < 0.05).

### 3.3. Moxibustion Reduced Neuronal Apoptosis

The neuronal apoptosis induced by cerebral ischemia/reperfusion was examined by terminal deoxynucleotidyl transferase-mediated dUTP nick end labeling (TUNEL), which selectively labels apoptotic cells. Apoptotic cells were stained green by TUNEL, while normal cells were stained blue by DAPI. The results showed that there was no obvious apoptosis in the brain tissue of the control group, and the cells in the brain tissue sections were mainly blue. In the I/R group, the number of green cells increased significantly, suggesting that I/R led to a significant increase in the number of apoptotic cells on the ischemic side of the brain. The apoptosis rate in the ischemic area was significantly higher than that in the control group (*P* < 0.001) (Figure 3).

Compared with that in the I/R group, the number of green cells in the I/R + Ro25-6981 group decreased, indicating that the number of apoptotic cells decreased and the apoptosis rate decreased (*P* < 0.001). Compared with I/R + Ro25-6981, after pretreatment with Ro25-6981 plus moxibustion, the number of green apoptotic cells decreased significantly, and the apoptosis rate decreased significantly (*P* < 0.001).

### 3.4. Moxibustion Upregulated the Protein Levels of Bcl-2 and Downregulated Bax and Caspase-3

After cerebral I/R injury, apoptosis-related factors are involved in the development of brain injury. Caspase-3 is involved in endogenous and exogenous apoptotic pathways. The Bcl-2 protein family is also involved in the process of apoptosis after cerebral ischemia, and there is a decrease in the antiapoptotic protein Bcl-2 and an increase in the proapoptotic protein Bax. The results showed that compared with the control group, the levels of caspase-3 and Bax in the I/R group increased significantly (*P* < 0.001), while the level of Bcl-2 decreased significantly (*P* < 0.001) (Figure 4).

Compared with the I/R group, the expression level of Bcl-2 in the I/R + moxibustion group increased significantly (*P* < 0.01), while the levels of caspase-3 and Bax decreased significantly (*P* < 0.001). Compared with the I/R group, the expression level of Bcl-2 in the I/R + Ro25-6981 group increased significantly (*P* < 0.001), while the levels of caspase-3 and Bax decreased significantly (*P* < 0.001). Compared with the I/R + Ro25-6981 group, the level of Bcl-2 in the I/R + moxibustion group increased more significantly (*P* < 0.05), and the expression level of caspase-3 decreased more significantly (*P* < 0.01). The level of Bax in the I/R + Ro25-6981 group decreased more significantly than that in the moxibustion group (*P* < 0.001).

### 3.5. Moxibustion Downregulated the Protein Levels of NR2B

NR2B is involved in the process of apoptosis in cerebral ischemia-reperfusion injury. The main subtypes of NMDA receptors include NR2A and NR2B. These subtypes play different roles in glutamate hyperstimulation. Excitotoxicity-dependent cell death is the result of overstimulation of NMDA receptors containing NR2B (rather than NR2A).

Figure 5 shows that compared with that in the control group, the gray value of NR2B in the I/R group increased, indicating that the expression of NR2B in brain tissue increased after I/R. The gray value of p-NR2B also increased significantly (*P* < 0.001), which indicated that the activity of NR2B increased significantly after I/R. Compared with that in the I/R group, the gray value of NR2B and p-NR2B in the I/R + moxibustion group decreased, indicating that the expression level of NR2B protein and activity of NR2B was downregulated after moxibustion treatment (*P* < 0.001). Compared with the I/R + moxibustion group, the gray value of NR2B and p-NR2B in the I/R + Ro25-6981 + moxibustion group decreased significantly, which indicated that the protein levels of NR2B and the activity of NR2B protein were downregulated significantly after Ro25-6981 + moxibustion treatment (*P* < 0.001).

### 3.6. Moxibustion Downregulated the Protein Levels of JNK

The c-Jun N-terminal kinase (JNK) signaling pathway plays an important role in cerebral ischemia/reperfusion injury and neuronal apoptosis. Cerebral ischemia/reperfusion activates the JNK signaling pathway, which can control the differential expression of apoptosis-related genes [27].

Figure 6(a) shows that compared with that in the control group, the gray value of JNK and p-JNK in the I/R group increased, which indicated that the protein level of JNK and the activity of JNK increased significantly after I/R ((*P* < 0.001). Compared with that in the I/R group, the gray value of JNK and p-JNK in the I/R + moxibustion group decreased, indicating that the expression level of JNK protein and activity of JNK were downregulated after moxibustion treatment (*P* < 0.001). Compared with the I/R + moxibustion group, the gray value of JNK increased and p-JNK decreased significantly in the I/R + Ro25-6981+moxibustion group, which indicated that the protein level of JNK increased (*P* < 0.05), but the activity of JNK protein was downregulated significantly after Ro25-6981 + moxibustion treatment (*P* < 0.001).

## 4. Discussion

The results of this study demonstrated that moxibustion can improve neurological dysfunction, decrease infarction area and neuronal apoptosis, downregulate the expression of NR2B and JNK, increase the level of Bcl-2, and decrease the level of caspase-3. Similarly, NR2B antagonist Ro25-6981 strengthened the improvements of neurological function, infarction area, neuronal apoptosis, and the changes of NR2B levels caused by I/R. Thus, moxibustion might exert a neuroprotective effect in the rat models of I/R injury by regulating the target of NR2B.

Nerve cell death and damage to the ischemic brain are a series of complicated pathological changes caused by limited blood flow in the ischemic area [28, 29]. Excitatory toxicity induced by the overexcitation of NMDA receptors is considered to be an important mechanism of apoptosis and brain injury after ischemia [30]. In the physiological state, NMDA receptors participate in high-level neural activities such as excitatory synaptic transmission, synaptic plasticity, learning, and memory, which are of great importance to the normal physiological activities of the nervous system [31]. Abnormal activation of NMDA receptors is important pathological pathogenesis of many nervous system diseases. NMDA receptors are gate-controlled ion channels. Among the NMDA receptor complexes, the subunits have been identified as NR1, NR2, and NR3, among which NR2 includes NR2A, NR2B, NR2C, NR2D, and other subunits. Among the various subunits of the NMDA receptor, NR2B is an important regulatory subunit [32]. Among these subunits, NR2A and NR2B have been widely studied because of their extensive expression in the brain [33]. In brain injury models such as cerebral ischemia, NR2A and NR2B participate in glutamate-mediated survival and death pathways in nerve cells, respectively. NR2B tends to promote neuronal death [12,34] while NR2A is associated with neuroprotection [9,35].

Activation of the c-Jun terminal kinase (JNK) signaling pathway is a key step in neuronal death in a variety of nervous system diseases and plays an important role in cerebral ischemia/reperfusion injury and neuronal apoptosis [36]. The JNK signaling pathway, also known as the stress-activated protein kinase signaling pathway, is an important component of serine protein kinase (MAPK) cascade activation. The MAPK signaling pathway plays an important role in the occurrence and development of cerebral ischemia [37]. Cerebral ischemia and hypoxia can activate MAPKs to regulate cell proliferation, differentiation, apoptosis, and other pathological changes, resulting in ischemic brain injury. The JNK signaling pathway is one of the three major MAPK pathways and is considered to be an important pathway for apoptosis. Activation of the JNK signaling pathway is a common factor in apoptosis induced by cerebral ischemia/reperfusion injury, oxidative stress, and inflammation [38,39]. Neuronal apoptosis induced by the JNK signaling pathway is related to the transcription and expression of bcl-2 gene family genes [40], especially Bcl-2 and Bax proteins [41]. The expression of Bcl-2 and Bax showed opposite trends. When the expression of Bcl-2 decreased and the expression of Bax increased, apoptosis was promoted, and when the expression of Bcl-2 increased and the expression of Bax decreased, apoptosis was inhibited [42]. The caspase family is the core of apoptosis, and active caspase-3 is the executor of apoptosis [43]. Caspase-3 induces a cascade reaction by cleaving other caspase substrates, which eventually leads to apoptosis. In this study, after cerebral ischemia-reperfusion, with the loss of neurological function, the increase of cerebral infarction area and neuronal apoptosis rate, the expression of NR2B and JNK increased, Bax and caspase-3 increased, and Bcl-2 decreased. This finding is consistent with the results of previous studies [38].

JNKs can be activated through receptor tyrosine kinases, cytokine receptors, G protein-coupled receptors, and ligand-gated ion channels, including NMDA glutamate receptors [44]. Studies have shown that NMDA receptors are related to the activation of JNK, and glutamate can increase the level of p-JNK in primary nerve cells [45]. NMDA receptors (NR1 and NR2B) act as upstream molecules of JNK signaling and Akt signaling, inducing JNK activation and weakening Akt activation in ischemic brain injury [46]. The selective noncompetitive NMDA glutamate receptor antagonist MK-801 almost completely blocks glutamate- and NMDA-induced JNK activation [47]. NR2B antagonists have protective effects on LPS-induced JNK phosphorylation in the frontal lobe and hippocampus [48]. The activation of NMDAR, especially NMDAR containing NR2B, plays a key role in the phosphorylation of JNK in astrocytes [49]. In this study, we found that the activation of JNK during a cerebral ischemia-reperfusion injury was related to NR2B. However, it should be noted that the NR2B antagonist Ro25-6981 could not completely block the activation of JNK. Therefore, the activation of JNK in nerve cells does not completely depend on NR2B. Other factors, such as cytokines and proinflammatory cytokines, may also play a role in the JNK pathway in cerebral ischemia-reperfusion injury.

Previous studies have shown that moxibustion has a neuroprotective effect on cerebral ischemic injury [24]. In this study, the GV20 acupoint located in the head and the GV14 acupoint in the neck were selected. These two acupoints are commonly used in neuroprotection mechanisms [23]. This study showed that Ro25-6981 could significantly inhibit the protein expression of NR2B and downregulate JNK in ischemia/reperfusion rats. Moxibustion could also significantly downregulate the protein expression of NR2B and JNK in I/R rats.

In this study, our results show that moxibustion can reduce NDS, cerebral infarction rate, and neuronal apoptosis induced by cerebral I/R in rats. Moxibustion can upregulate the level of Bcl-2 protein and downregulate the levels of Bax, caspase-3, and JNK protein. Its effect is similar to that of NR2B antagonist Ro25-6981, suggesting that moxibustion may be an effective neuroprotective measure for the treatment of ischemic stroke. The study suggests that the neuroprotective mechanism of moxibustion is related to downregulating the expression of NR2B, in which the JNK signal pathway plays an important role. Moxibustion has a better effect of downregulating JNK than Ro25-6981, so the effect of downregulating JNK by moxibustion may not only be realized by downregulating NR2B, but we need to further explore in future research.

## 5. Conclusion

Moxibustion can improve neurological dysfunction and decrease infarction area and neuronal apoptosis caused by cerebral ischemia/reperfusion in rats. Its neuroprotective mechanism may be related to downregulating the expression of NR2B.

## 6. Ethics Approval

The animal study was reviewed and approved by the Institutional Animal Care and Use Committee of Zhejiang Chinese Medical University.

## Figures and Tables

**Figure 1:** Neurological deficit score.

**Figure 2:** TTC staining of rat brain tissue in each group. (a) TTC staining of brain tissue in each group. The pink area is normal brain tissue, and the pale area is the ischemic infarcted area. (b) Cerebral infarction rates of rats in each group. ^*∗*^*P* < 0.05 and ^*∗∗∗*^*P* < 0.001 compared to the control group; ^##^*P* < 0.01 and ^###^*P* < 0.001 versus the I/R group; ^※^*P* < 0.05 versus the I/R + Ro25-6981 group.

**Figure 3:** TUNEL staining of rat brain tissue in each group. (a) TUNEL staining results of brain tissue in each group. TUNEL staining showed green apoptotic cells while DAPI staining showed blue normal cells. The merged images included green apoptotic cells and blue normal cells. (b) Statistical analysis of the apoptosis rate on the injured side of the brain in each group. ^*∗∗*^*P* < 0.01 and ^*∗∗∗*^*P* < 0.001 compared to the control group; ^###^*P* < 0.001 versus the I/R group; ^△△△^*P* < 0.001 versus the I/R + moxibustion group; ^※※※^*P* < 0.001 versus the I/R + Ro25-6981 group.

**Figure 4:** Analysis of the relative expression of apoptosis-related proteins in brain tissue in each group. (a) Protein expression of cleaved caspase-3, Bcl-2, and Bax on the ischemic side in each group. (b) Relative protein expression of Bcl-2, Bax, and cleaved caspase-3 on the ischemic side in each group. ^*∗∗∗*^*P* < 0.001 compared to the control group; ^##^*P* < 0.01 and ^###^*P* < 0.001 versus the I/R group; ^△^*P* < 0.05, ^△△^*P* < 0.01, and ^△△△^*P* < 0.001 versus the I/R + moxibustion group; ^※※※^*P* < 0.001 versus the I/R+ Ro25-6981 group.

**Figure 5:** Relative expression of NR2B and p-NR2B protein in brain tissue of each group. (a) Protein expression of NR2B and p-NR2B in the injured brain tissue of each group. (b) Relative protein expression levels of NR2B and p-NR2B in the injured brain tissue of each group. ^*∗∗∗*^*P* < 0.001 compared to the control group; ^###^*P* < 0.001 versus the I/R group; ^△△△^*P* < 0.001 versus the I/R + moxibustion group; ^※※※^*P* < 0.001 versus the I/R + Ro25-6981 group.

**Figure 6:** Relative protein expression of JNK and p-JNK in the brain tissues in the different groups. (a) Protein expression of JNK and p-JNK in the injured brain tissue of each group. (b) Relative protein expression levels of JNK and p-JNK in the injured brain tissue of each group. ^*∗∗∗*^*P* < 0.001 compared to the control group; ^###^*P* < 0.001 versus the I/R group; ^△^*P* < 0.05 and ^△△△^*P* < 0.001 versus the I/R + moxibustion group; ^※※※^*P* < 0.001 versus the I/*R* + Ro25-6981 group.

## Data Availability

The raw data supporting the conclusions of this article will be made available by the authors, without undue reservation.
